The article "Classical and Bayesian Inference Using Type-II Unified Progressive Hybrid Censored Samples for Pareto Model" was published in 2022. Journal: Appl Bionics Biomech.

# Classical and Bayesian Inference Using Type-II Unified Progressive Hybrid Censored Samples for Pareto Model

**DOI:** 10.1155/2022/2073067

**Published:** 2022-04-29

**Authors:** M. Nagy, Adel Fahad Alrasheedi

**Affiliations:** Department of Statistics and Operations Research, College of Science, King Saud University, P.O. Box 2455, Riyadh 11451, Saudi Arabia

## Abstract

In the lifetime and reliability experiments, the censored samples play a fundamental and important role in order to control time and cost. The researchers developed the censored sample schemes to solve the problems that arise by applying the previous methods. Recently, Górny and Cramer (2018) proposed a new general type of censored sample called Type-II unified progressive hybrid censored sample. In this paper, we present an overview of the Type-II unified progressive hybrid censored sample. We used this censored sample to compute the maximum likelihood estimates of unknown parameters from the Pareto distribution, as well as Bayesian estimates for unknown parameters under three different error loss functions. The point and interval Bayesian predictions one- and two-sample Bayesian predictions from the Pareto distribution are shown. Simulation studies are carried out to compare the efficacy of the various inference approaches. Finally, real data sets are examined to determine the applicability of the proposed model and various estimating approaches.

## 1. Introduction

In order to time and expense constraints, experiments in reliability analysis frequently end before all units in the test have failed. In such circumstances, failure information is only accessible for a portion of the sample, and only limited information is given on all units that have not failed. Data that has been censored is referred to as censored data. There are several different censoring schemes such as Type-I and Type-II. Since Epstein [1] presented Type-I hybrid censoring, various hybrid censoring modifications have been developed to address the model's flaws. Due to the fact that Type-I hybrid censoring does not guarantee the observation of at least one of the failures, Childs et al. [2] developed Type-II hybrid censoring, which ensures the observation of at least *m* failures from the *n* units put on the life test. However, the main disadvantage of this censoring system is that the experimenter has not controlled the test time. The disadvantages of both Type-I and Type-II hybrid censoring are mitigated by Chandrasekar et al. [3]. In addition, the unified hybrid censoring methods are even more flexible than hybrid censoring techniques (see, e.g., Balakrishnan et al. [4]; Huang and Yang [5]; Park and Balakrishnan [6]). In unified hybrid censoring method, consider, *n* identical units are placed on a life-testing device. Fix the integers *k*, *m* ∈ {1, 2, ⋯, *n*}, and *T*_1_ and *T*_2_∈(0, ∞) such that *k* < *m* and *T*_1_ < *T*_2_. The experiment is stopped at min(max(*T*_1_, *Y*_*m*:*n*_), *T*_2_) if the *k*^th^ failure occurs before time *T*_1_. Otherwise, the experiment is stopped at min(max(*Y*_*k*:*n*_, *T*_2_), *Y*_*m*:*n*_)%. We can guarantee that the experiment will be completed at most in time *T*_2_ with at least *k* failures, and if not, we can guarantee exactly *k* failures under this censoring strategy.

If one of these units is inadvertently broken but the experiment has not yet been terminated, this unit must be removed from the life test, and the progressive censoring methodology is the best method for this case. Complete failures of *m* units will be observed in Type-II progressive censoring methods. When the first failure occurs, *R*_1_ of the *n* − 1 remaining units is chosen at random and removed from the lifetime test. *R*_2_ of the *n* − *R*_1_ − 2 surviving units is randomly selected and eliminated at the second observed failure. Finally, *R*_*m*_ surviving units are removed after the *m*^th^ failure, and the experiment comes to an end. We will denote the *m* ordered failure times thus observed by *Y*_1:*m*:*n*_, ⋯, *Y*_*m*:*m*:*n*_. It is evident that *n* = *m* + ∑_*k*=1_^*m*^*R*_*k*_.

The downsides of the Type-II progressive censoring system are that if the units are highly reliable, the experiment can take a long time. Therefore, Kundu and Joarder [7] and Childs et al. [8] proposed a progressive hybrid censoring scheme (PHCS) in which the life-testing experiment is ended at time min{*Y*_*m*:*m*:*n*_, *T*}, with *T* ∈ (0, ∞). For more details, we refer our readers to Tomer and Panwar [9], Panahi [10], Almarashi et al. [11], and Moihe El-Din et al. [12, 13]. On the other hand, the disadvantage of the PHCS is that it cannot be applied when only a few failures are likely to occur before time *T*. For this reason, Cho et al. [14] proposed a Type-I generalized PHCS in which the life-testing experiment is terminated at the time min{max(*T*, *Y*_*k*:*m*:*n*_), *Y*_*m*:*m*:*n*_} for prefixed *k* < *m*{1, 2, ⋯, *n*}. Moreover, Lee et al. [15] proposed Type-II generalized PHCS, in which the life-testing experiment is terminated at time min{max(*T*_1_, *Y*_*m*:*m*:*n*_), *T*_2_} for prefixed *T*_1_ < *T*_2_(0, ∞). For recent work on this topic, see, for example, Moihe El-Din and Nagy [16], Nagy et al. [17, 18], and Nagy and Alrasheedi [19].

While generalized PHCS are superior to Type-I and Type-II PHSC, they do have significant disadvantages. Therefore, Górny and Cramer [20] developed a general type of generalized PHCS, called Type-II unified PHCS to address some of the shortcomings of these schemes. Under Type-II unified PHCS, we can guarantee that the lifetime experiment will be completed at no later than *T*_2_ with at least *k* number of unit failures; this ensures that the statistical inference is carried out with more efficiency. For recent work on the Type-II unified PHCS, see, for example, Górny and Cramer in [21] and Kim and Lee in [22].

The following is how the rest of the article is structured: Section 2 provides an overview of the Type-II unified PHCS.  Section 3 determines the maximum likelihood estimates (ML) of unknown parameters, while Section 4 derives the Bayesian estimates for the unknown parameters with three loss functions. Sections 5 and 6 calculate the point and interval Bayesian predictions for one- and two-sample Bayesian predictions, respectively. Simulation studies are carried out in Section 7 to compare the efficacy of the offered inference methodologies. A real data is utilized to demonstrate the theoretical findings in Section 8. Finally, the paper is concluded in Section 9.

## 2. The Type-II Unified PHCS and Likelihood Function

Consider a life test in which *n* identical items are put on test. Then, the Type-II unified PHCS may be described as follows. Let *T*_1_, *T*_2_ ∈ (0, ∞) and integer *k*, *m* ∈ {1, 2, ⋯, *n*} are prefixed such that *T*_1_ < *T*_2_ and *k* < *m* with *R* = (*R*_1_, *R*_2_, ⋯, *R*_*m*_) is also prefixed integers satisfying *n* = *m* + *R*_1_ + ⋯+*R*_*m*_. At the time of first failure, *R*_1_ of the remaining units are randomly removed. Similarly, at the time of the second failure *R*_2_, of the remaining units are removed and so on. If the *k*^th^ failure occurs before time *T*_1_, the experiment is terminated at min{max(*Y*_*m*:*m*:*n*_, *T*_1_), *T*_2_}. If the *k*^th^ failure occurs between *T*_1_ and *T*_2_, the experiment is terminated at min(*Y*_*rm*:*m*:*n*_, *T*_2_) and if the *k*^th^ failure occurs after time *T*_2_, the experiment is terminated at *Y*_*k*:*n*_. Under this censoring scheme, we can guarantee that the experiment would be completed at most in time *T*_2_ with at least *k* failure and if not, we can guarantee exactly *k* failures. Let *D*_1_ and *D*_2_ denote the numbers of observed failures up to time *T*_1_ and *T*_2_, respectively. In addition, *d*_1_ and *d*_2_ are the observed values of *D*_1_ and *D*_2_, respectively.

Under the UPHCS described above, we have one of the following types of observations:

1. If the *k*^th^ failure occurs before time *T*_1_, the experiment is terminated at min{max(*Y*_*m*:*m*:*n*_, *T*_1_), *T*_2_} and then we have the following three subcases:

- If the *m*^th^ failure occurs before *T*_1_, i.e., 0 < *Y*_*k*:*m*:*n*_ < *Y*_*m*:*m*:*n*_ < *T*_1_ < *T*_2_, then instead of terminating the test by withdrawing the remaining *R*_*m*_ items after the *m*^th^ failure, we continue to observe failures (without any further withdrawals) up to the experiment end at time *T*^∗^ = *T*_1_. Therefore, the observed failure times are {*Y*_1:*m*:*n*_<⋯<*Y*_*k*:*m*:*n*_<⋯<*Y*_*m*:*m*:*n*_<⋯<*Y*_*d*_1_:*n*_}
- If the *m*^th^ failure occurs between *T*_1_ and *T*_2_, i.e., 0 < *Y*_*k*:*m*:*n*_ < *T*_1_ < *Y*_*m*:*m*:*n*_ < *T*_2_, then the experiment will end at *T*^∗^ = *Y*_*m*:*m*:*n*_ and the observed failure times are {*Y*_1:*m*:*n*_<⋯<*Y*_*k*:*m*:*n*_<⋯<*Y*_*d*_1_:*m*:*n*_<⋯<*Y*_*m*:*m*:*n*_}
- If the *m*^th^ failure occurs after *T*_2_, i.e., 0 < *Y*_*k*:*m*:*n*_ < *T*_1_ < *T*_2_ < *Y*_*m*:*m*:*n*_, then the experiment will end at *T*^∗^ = *T*_2_ and the observed failure times are {*Y*_1:*m*:*n*_<⋯<*Y*_*k*:*m*:*n*_<⋯<*Y*_*d*_1_:*m*:*n*_<⋯<*Y*_*d*_2_:*m*:*n*_}

(2) If the time *T*_1_ pass before the *k*^th^, then the experiment will end at min{max(*Y*_*k*:*m*:*n*_, *T*_2_), *Y*_*m*:*m*:*n*_} and then we have the following three subcases:
  - If *T*_2_ passes before the *k*^th^ failure occurs, i.e., 0 < *T*_1_ < *T*_2_ < *Y*_*k*:*m*:*n*_ < *Y*_*m*:*m*:*n*_, then the experiment will end at *T*^∗^ = *Y*_*k*:*m*:*n*_ and we will observe {*Y*_1:*m*:*n*_<⋯<*Y*_*d*_1_:*m*:*n*_<⋯<*Y*_*d*_2_:*m*:*n*_<⋯<*Y*_*k*:*m*:*n*_}
  - If the *m*^th^ failure occurs before *T*_2_, i.e., 0 < *T*_1_ < *Y*_*k*:*m*:*n*_ < *Y*_*m*:*m*:*n*_ < *T*_2_, then the experiment will end at *T*^∗^ = *Y*_*m*:*m*:*n*_ and we will observe {*Y*_1:*m*:*n*_<⋯<*Y*_*d*_1_:*m*:*n*_<⋯<*Y*_*k*:*m*:*n*_<⋯<*Y*_*m*:*m*:*n*_}
  - If the time *T*_2_ between *Y*_*k*:*m*:*n*_ and *Y*_*m*:*m*:*n*_, i.e., 0 < *T*_1_ < *Y*_*k*:*m*:*n*_ < *T*_2_ < *Y*_*m*:*m*:*n*_, then the experiment will end at *T*^∗^ = *T*_2_ and the observed failure times are {*Y*_1:*m*:*n*_<⋯<*Y*_*d*_1_:*m*:*n*_<⋯<*Y*_*k*:*m*:*n*_<⋯<*Y*_*d*_2_:*m*:*n*_}

Let $\underline{Y}$ be the Type-II unified progressive hybrid censored sample from distribution with the probability density function (PDF) *g*(*y*), and the cumulative distribution function (CDF) *G*(*y*), then, based on the Type-II unified PHCS, the likelihood function is given by

(1) $$\begin{array}{c} L_{\underline{Y}}\left(\underline{Y}\right)=\left\{\begin{array}{cc} \left[\overset{d_{1}}{\underset{i=1}{\prod }}\overset{m}{\underset{j=1}{\sum }}\left({\tilde{R}}_{j}+1\right)\right]\overset{d_{1}}{\underset{i=1}{\prod }}g\left(y_{i:m:n}\right){\left[\bar{G}\left(y_{i:m:n}\right)\right]}^{{\tilde{R}}_{i}}{\left[\bar{G}\left(T_{1}\right)\right]}^{{\tilde{R}}_{t_{1}}} & \text{in Case }1_{a},\\ \left[\overset{m}{\underset{i=1}{\prod }}\overset{m}{\underset{j=1}{\sum }}\left({\tilde{R}}_{j}+1\right)\right]\overset{m}{\underset{i=1}{\prod }}g\left(y_{i:m:n}\right){\left[\bar{G}\left(y_{i:m:n}\right)\right]}^{{\tilde{R}}_{i}} & \text{in Case }1_{b},\\ \left[\overset{d_{2}}{\underset{i=1}{\prod }}\overset{m}{\underset{j=1}{\sum }}\left({\tilde{R}}_{j}+1\right)\right]\overset{d_{2}}{\underset{i=1}{\prod }}g\left(y_{i:m:n}\right){\left[\bar{G}\left(y_{i:m:n}\right)\right]}^{{\tilde{R}}_{i}}{\left[\bar{G}\left(T_{2}\right)\right]}^{{\tilde{R}}_{t_{2}}} & \text{in Case }1_{c},\\ \left[\overset{k}{\underset{i=1}{\prod }}\overset{m}{\underset{j=1}{\sum }}\left({\tilde{R}}_{j}+1\right)\right]\overset{k}{\underset{i=1}{\prod }}g\left(y_{i:m:n}\right){\left[\bar{G}\left(y_{i:m:n}\right)\right]}^{{\tilde{R}}_{i}} & \text{in Case }2_{a},\\ \left[\overset{m}{\underset{i=1}{\prod }}\overset{m}{\underset{j=1}{\sum }}\left({\tilde{R}}_{j}+1\right)\right]\overset{m}{\underset{i=1}{\prod }}g\left(y_{i:m:n}\right){\left[\bar{G}\left(y_{i:m:n}\right)\right]}^{{\tilde{R}}_{i}} & \text{in Case }2_{b},\\ \left[\overset{d_{2}}{\underset{i=1}{\prod }}\overset{m}{\underset{j=1}{\sum }}\left({\tilde{R}}_{j}+1\right)\right]\overset{d_{2}}{\underset{i=1}{\prod }}g\left(y_{i:m:n}\right){\left[\bar{G}\left(y_{i:m:n}\right)\right]}^{{\tilde{R}}_{i}}{\left[\bar{G}\left(T_{2}\right)\right]}^{{\tilde{R}}_{t_{2}}} & \text{in Case }2_{c}, \end{array}\right. \end{array}$$

Therefore, these cases can be combined and obtained as

(2) $$\begin{array}{c} L\left(\theta \;|\;\underline{Y}\right)\left[\overset{d^{*}}{\underset{i=1}{\prod }}\overset{m}{\underset{j=1}{\sum }}\left({\tilde{R}}_{j}+1\right)\right]\overset{d^{*}}{\underset{i=1}{\prod }}g\left(y_{i:m:n}\right){\left[\bar{G}\left(y_{i:m:n}\right)\right]}^{{\tilde{R}}_{i}}{\left[\bar{G}\left(T_{1}\right)\right]}^{{\tilde{R}}_{t_{1}}}{\left[\bar{G}\left(T_{2}\right)\right]}^{{\tilde{R}}_{t_{2}}}, \end{array}$$

where $\bar{G}=1-G$ and

(3) $$\begin{array}{c} \underline{Y}=\left\{\begin{array}{cc} \left(y_{1:m:n},\cdots ,y_{k:m:n},\cdots ,y_{m-1:m:n},y_{m:m:n},\cdots ,y_{d1:n}\right) & \text{in Case }1_{a},\\ \left(y_{1:m:n},\cdots ,y_{k:m:n},\cdots ,y_{d1:m:n},\cdots ,y_{m:m:n}\right) & \text{in Case }1_{b},\\ \left(y_{1:m:n},\cdots ,y_{k:m:n},\cdots ,y_{d1:m:n},\cdots ,y_{d2:m:n}\right) & \text{in Cases }1_{c},\\ \left(y_{1:m:n},\cdots ,y_{d1:m:n},\cdots ,y_{d2:m:n},\cdots ,y_{k:m:n}\right) & \text{in Case }2_{a},\\ \left(y_{1:m:n},\cdots ,y_{d_{1}},\cdots ,y_{k:m:n},\cdots ,y_{m:m:n}\right) & \text{in Case }2_{b},\\ \left(y_{1:m:n},\cdots ,y_{d1:m:n},\cdots ,y_{k:m:n},\cdots ,y_{d2:m:n}\right) & \text{in Cases }2_{c}, \end{array}\right.\\ d^{*}=\left\{\begin{array}{cc} d_{1} & \text{in Case }1_{a},\\ m & \text{in Cases }1_{b}\text{ and }2_{b},\\ d_{2} & \text{in Cases }1_{c}\text{ and }2_{c},\\ k & \text{in Case }2_{a}, \end{array}\right.\\ \tilde{R}=\begin{array}{cc} \left(R_{1},\cdots ,R_{k},\cdots ,R_{m-1},0,\cdots ,0,R_{t_{1}}\right) & \text{in Case }1_{a},\\ \left(R_{1},\cdots ,R_{k},\cdots ,R_{d_{1}},\cdots ,R_{m}\right) & \text{in Case }1_{b},\\ \left(R_{1},\cdots ,R_{k},\cdots ,R_{d_{1}},\cdots ,R_{t_{2}}\right) & \text{in Cases }1_{c},\\ \left(R_{1},\cdots ,R_{d_{1}},\cdots ,R_{d_{2}},\cdots ,R_{k^{*}}\right) & \text{in Case }2_{a},\\ \left(R_{1},\cdots ,R_{d_{1}},\cdots ,R_{k},\cdots ,R_{m}\right) & \text{in Case }2_{b},\\ \left(R_{1},\cdots ,R_{d_{1}},\cdots ,R_{k},\cdots ,R_{t_{2}}\right) & \text{in Cases }2_{c}, \end{array} \end{array}$$

with ${\tilde{R}}_{k^{*}}=n-k-\sum_{j=1}^{k-1}{\tilde{R}}_{j},$${\tilde{R}}_{t_{1}}$ is the number of surviving units that are eliminated at *T*_1_, given by

(4) $$\begin{array}{c} {\tilde{R}}_{t_{1}}=\left\{\begin{array}{cc} n-d_{1}-\overset{m-1}{\underset{j=1}{\sum }}{\tilde{R}}_{j} & \text{in Case }1_{a},\\ 0 & \text{in all other cases}, \end{array}\right. \end{array}$$

and ${\tilde{R}}_{t_{2}}$ is the number of surviving units that are eliminated at *T*_2_, given by

(5) $$\begin{array}{c} {\tilde{R}}_{t_{2}}=\left\{\begin{array}{cc} n-d_{2}-\overset{d_{2}}{\underset{j=1}{\sum }}{\tilde{R}}_{j} & \text{in Cases }1_{c}\text{ and }2_{c},\\ 0 & \text{in all other cases}. \end{array}\right. \end{array}$$

Special cases: The Type-II unified PHCS is a generalization of many censoring schemes, for example:

1. If *R*_*i*_ = 0 for all *i* < *m* and *R*_*m*_ = *n* − *m*, the Type-II unified PHCS becomes unified HCS
2. If *T*_2_ = ∞, the Type-II unified PHCS becomes generalized Type-I PHCS
3. If *k* = *m*, the Type-II unified PHCS becomes generalized Type-II PHCS
4. If *T*_1_ = 0 and *k* = *m*, the Type-II unified PHCS becomes Type-I PHCS
5. If *T*_2_ = ∞ and *k* = 0, the Type-II unified PHCS becomes Type-II PHCS

**Note:** In order for the experiment to be terminated at time *T*_1_, *R*_*m*_ must be not equal to zero; if *R*_*m*_ is equal to zero and the *m*^th^ failure occurs before *T*_1_, then the experiment is terminated at *Y*_*m*:*m*:*n*_.

## 3. The ML Estimation

In this section, we derive the ML inference of the unknown parameters *λ* and *θ* for the Pareto distribution which was introduced by Pareto [23] as a model for the distribution of income, based on the Type-II unified PHCS. Using the exponential form, Pareto distribution has the following density function (PDF) and distribution function (CDF), respectively, given by

(6) $$\begin{array}{c} g\left(y\;|\;\lambda ,\theta \right)=\frac{\lambda }{y}\exp\left[-\lambda \ln\left(\frac{y}{\theta }\right)\right],\lambda ,\theta >0,y\geq \theta , \end{array}$$

(7) $$\begin{array}{c} G\left(y\;|\;\lambda ,\theta \right)=1-\exp\left[-\lambda \ln\left(\frac{y\%}{\theta }\right)\right],\lambda ,\theta >0,y\geq \theta .\%. \end{array}$$

From (7), (6), and (2), the likelihood function of *λ*, *θ* under the Type-II unified PHCS can be derived as

(8) $$\begin{array}{c} L\left(\lambda ,\theta \;|\;\underline{Y}\right)=\left[\overset{d^{*}}{\underset{i=1}{\prod }}\overset{m}{\underset{j=i}{\sum }}\left(\;{\tilde{R}}_{j}+1\right)\right]\lambda^{d^{*}}\left(\underset{i=1}{\prod^{d^{*}}}\frac{1}{y_{i}}\right)\exp\left\{-\lambda \left[\eta \left(\underline{y}\right)+{\tilde{R}}_{t_{1}}\ln T_{1}+{\tilde{R}}_{t_{2}}\ln T_{2}-n\ln\theta \right]\right\}, \end{array}$$

where $\eta \left(\underline{y}\right)=\sum_{i=1}^{d^{*}}\left({\tilde{R}}_{i}+1\right)\ln y_{i}$, and *y*_*i*_ = *y*_*i*:*d*^∗^:*n*_ for simplicity of notation.

Since the likelihood function (8) is an increasing function in *θ*, but *θ* is the lower bound of *y*_*i*_ for all $y_{i}\in \underline{Y}$, so its maximum value will be attained at the maximum value *y*_1_ of *θ*. From (8), the log-likelihood function of (*λ*, *θ*) is given by

(9) $$\begin{array}{c} \ln\left[L\left(\lambda ,\theta \;|\;\underline{Y}\right)\right]\propto d^{*}\ln\left(\lambda \right)-\lambda \left[\eta \%\left(\underline{y}\right)+{\tilde{R}}_{t_{1}}\ln T_{1}+{\tilde{R}}_{t_{2}}\ln T_{2}-n\ln\left(\theta \right)\right]. \end{array}$$

To maximize relative to *λ*, differentiate (9) with respect to *λ* and solve the equation

(10) $$\begin{array}{c} \frac{\partial \ln\left[L\left(\lambda ,\theta \;|\;\underline{Y}\right)\right]}{\partial \lambda }=0, \end{array}$$

so the ML estimator ${\hat{\lambda }}_{ML}$ of *λ* is obtained as

(11) $$\begin{array}{c} {\hat{\lambda }}_{ML}=\frac{d^{*}}{\eta \left(\underline{y}\right)+{\tilde{R}}_{t_{1}}\ln T_{1}+{\tilde{R}}_{t_{2}}\ln T_{2}-n\ln\left(y_{1:n}\right)}. \end{array}$$

### 3.1. Approximate Confidence Intervals for *λ* and *θ*

For large *d*^∗^, the observed Fisher information matrix of the parameters *λ* and *θ* is given by

(12) $$\begin{array}{c} I\left(\hat{\lambda },\hat{\theta }\right)={\left[\begin{array}{cc} -\frac{\partial^{2}\ln L\left(\lambda ,\theta \;|\;\underline{Y}\right)}{\partial \lambda^{2}} & -\frac{\partial^{2}\ln L\left(\lambda ,\theta \;|\;\underline{Y}\right)}{\partial \lambda \partial \theta }\\ -\frac{\partial^{2}\ln L\left(\lambda ,\theta \;|\;\underline{Y}\right)}{\partial \theta \partial \lambda } & -\frac{\partial^{2}\ln L\left(\lambda ,\theta \;|\;\underline{Y}\right)}{\partial \theta^{2}} \end{array}\right]}_{\left({\hat{\lambda }}_{ML},{\hat{\theta }}_{ML}\right)}, \end{array}$$

where

(13) $$\begin{array}{c} \begin{array}{c} \frac{\partial^{2}\ln L\left(\lambda ,\theta \;|\;\underline{Y}\right)}{\partial \lambda^{2}}=-\frac{d^{*}}{\lambda^{2}},\\ \frac{\partial^{2}\ln L\left(\lambda ,\theta \;|\;\underline{Y}\right)}{\partial \theta^{2}}=-\frac{n\lambda }{\theta^{2}},\\ \frac{\partial^{2}\ln L\left(\lambda ,\theta \;|\;\underline{Y}\right)}{\partial \lambda \partial \theta }=-\frac{n}{\theta }, \end{array} \end{array}$$

and a 100(1 − *α*)% two-sided approximate confidence intervals for the parameters *λ* and *θ* are then

(14) $$\begin{array}{c} \left(\hat{\lambda }-z_{\alpha /2}\sqrt{V\left(\hat{\lambda }\right)},\hat{\lambda }+z_{\alpha /2}\sqrt{V\left(\hat{\lambda }\right)}\right),\\ \left(\hat{\theta }-z_{\alpha /2}\sqrt{V\left(\hat{\theta }\right)},\hat{\theta }+z_{\alpha /2}\sqrt{V\left(\hat{\theta }\right)}\right), \end{array}$$

respectively, where $V\left(\hat{\lambda }\right)$ and $V\left(\hat{\theta }\right)\;$ are the estimated variances of ${\hat{\lambda }}_{ML}$ and ${\hat{\theta }}_{ML}$, which are given by the first and the second diagonal element of $I^{-1}\left(\hat{\lambda },\hat{\theta }\right)$, and *z*_*α*/2_ is the upper (*α*/2) percentile of the standard normal distribution.

## 4. Bayesian Estimation

In this study, we investigate three forms of loss functions for Bayesian estimation. The first is the squared error loss function (SELF), which is a symmetric function that values overestimation and underestimation equally when estimating parameters. The LINEX loss function (LLF), which is asymmetric and offers different weights due to overestimation and underestimation, is the second option. The generalization of the entropy loss function is the third loss function (GELF).

Under the assumption that both parameters *λ* and *θ* are unknown, we can use the joint prior density function of *λ* and *θ* proposed by Lwin [24] and generalized by Arnold and Press [25] for Bayesian Estimations. The generalized Lwin prior is given by

(15) $$\begin{array}{c} \pi \left(\lambda ,\theta \right)\propto \frac{\lambda^{a_{1}}}{\theta }\exp\left[-\lambda \left(\ln a_{2}-b_{1}\ln\theta \right)\right],\lambda >0,0<\theta <d, \end{array}$$

where *a*_1_, *b*_1_, *a*_2_, *b*_2_ are positive constants and *b*_2_^*b*_1_^ < *a*_2_.

Upon combining (8) and (15), given UPHCS, the posterior density function of *λ*, *θ* is obtained as

(16) $$\begin{array}{c} \pi^{*}\left(\lambda ,\theta \;|\;\underline{Y}\right)=\frac{L\left(\lambda ,\theta \;|\;\underline{Y}\right)\pi \left(\lambda ,\theta \right)}{\int_{0}^{\infty }L\left(\lambda ,\theta \;|\;\underline{Y}\right)\pi \left(\lambda ,\theta \right)d\lambda d\theta }=I^{-1}\lambda^{d^{*}+a_{1}}\theta^{-1}\exp\left\{\left[-\lambda \eta \left(\underline{y}\right)+{\tilde{R}}_{t_{1}}\ln T_{1}+{\tilde{R}}_{t_{2}}\ln T_{2}-\left(n+b_{1}\right)\ln\theta +\ln a_{2}\right]\right\}, \end{array}$$

where

(17) $$\begin{array}{c} I=\int_{0}^{\delta }\int_{0}^{\infty }\lambda^{d^{*}+a_{1}}\theta^{-1}\exp\left\{-\lambda \left[\eta \left(\underline{y}\right)+{\tilde{R}}_{t_{1}}\ln T_{1}+{\tilde{R}}_{t_{2}}\ln T_{2}-\left(n+b_{1}\right)\ln\theta +\ln a_{2}\right]\right\}d\lambda d\theta =\frac{\Gamma \left(d^{*}+a_{1}\right)}{n+b_{1}}{\left[\eta \left(\underline{y}\right)+{\tilde{R}}_{t_{1}}\ln T_{1}+\tilde{R}{}_{t_{2}}\ln T_{2}-\left(n+b_{1}\right)\ln\delta +\ln a_{2}\right]}^{-\left(d^{*}+a_{1}\right)}, \end{array}$$

with *δ* = min(*y*_1:*n*_, *b*_2_).

### 4.1. The Bayesian Estimation under SELF

A commonly used loss function is the squared error loss function (SELF) defined as follows:

(18) $$\begin{array}{c} L_{BS}\left(\hat{\beta },\beta \right)\propto {\left(\overset{\wedge }{\beta }-\beta \right)}^{2} \end{array}$$

The Bayesian estimate ${\hat{\beta }}_{BS}$ for the unknown parameter *β*, relative to the squared error loss function, is given by

(19) $$\begin{array}{c} {\hat{\beta }}_{BS}=E_{\pi^{*}}\left[\beta \right] \end{array}$$

By using (16), the Bayesian estimator of *λ* under the squared error loss function is the mean of the posterior density function, given by

(20) $$\begin{array}{c} {\hat{\lambda }}_{BS}=\int_{0}^{\delta }\int_{0}^{\infty }\lambda \pi^{*}\left(\lambda ,\theta \;|\;\underline{Y}\right)d\lambda d\theta . \end{array}$$

Hence, the Bayesian estimator of *λ* under the squared error loss function is obtained as

(21) $$\begin{array}{c} {\hat{\lambda }}_{BS}=\frac{d^{*}+a_{1}}{\eta \left(\underline{y}\right)+{\tilde{R}}_{t_{1}}\ln T_{1}+{\tilde{R}}_{t_{2}}\ln T_{2}-\left(n+b_{1}\right)\ln\delta +\ln a_{2}}, \end{array}$$

and the Bayesian estimator of *θ* under the squared error loss function is obtained as

(22) $$\begin{array}{c} {\hat{\theta }}_{BS}=\int_{0}^{\delta }\int_{0}^{\infty }\theta \pi^{*}\left(\lambda ,\theta \;|\;\underline{Y}\right)d\lambda d\theta =I^{-1}\delta \int_{0}^{\infty }\frac{\lambda^{d^{*}+a_{1}}}{\lambda \left(n+b_{1}\right)+1}\exp\left\{-\lambda \left[\eta \left(\underline{y}\right)+{\tilde{R}}_{t_{1}}\ln T_{1}+{\tilde{R}}_{t_{2}}\ln T_{2}-\left(n+b_{1}\right)\ln\delta +\ln a_{2}\right]\right\}d\lambda =\frac{I^{-1}\delta }{\left(n+b_{1}\right)}{\left[\eta \left(\underline{y}\right)+{\tilde{R}}_{t_{1}}\ln T_{1}+{\tilde{R}}_{t_{2}}\ln T_{2}-\left(n+b_{1}\right)\ln\delta +\ln a_{2}\right]}^{-\left(d^{*}+a_{1}\right)}\times \int_{0}^{\infty }\frac{t^{d^{*}+a_{1}}e^{-t}}{t+\left[\eta \left(\underline{y}\right)+{\tilde{R}}_{t_{1}}\ln T_{1}+{\tilde{R}}_{t_{2}}\ln T_{2}-\left(n+b_{1}\right)\ln\delta +\ln a_{2}\right]/\left(n+b_{1}\right)}dt=\frac{\delta }{\Gamma \left(d^{*}+a_{1}\right)}\Phi \left(d^{*}+a_{1},\frac{\left[\eta \left(\underline{y}\right)+{\tilde{R}}_{t_{1}}\ln T_{1}+{\tilde{R}}_{t_{2}}\ln T_{2}-\left(n+b_{1}\right)\ln\delta +\ln a_{2}\right]}{\left(n+b_{1}\right)}\right), \end{array}$$

where

(23) $$\begin{array}{c} \Phi \left(y,y\right)=\int_{0}^{\infty }\frac{t^{y}e^{-t}}{t+y}dt. \end{array}$$

A partial tabulation of *ψ*(*y*, *y*) = (*y*/Γ(*y*))*Φ*(*y* − 1, *y*) has been provided by Arnold and Press in [25].

### 4.2. The Bayesian Estimation under GELF

Another commonly used asymmetric loss function is the general entropy (GE) loss function given by

(24) $$\begin{array}{c} L_{BE}\left(\hat{\beta },\beta \right)\propto {\left(\frac{\overset{\wedge }{\beta }}{\beta }\right)}^{\omega }-\omega \ln\left(\frac{\hat{\beta }}{\beta }\right)-1. \end{array}$$

For *ω* > 0, a positive error has a more serious effect than a negative error, and for *ω* < 0, a negative error has a more serious effect than a positive error. In this case, the Bayesian estimate ${\hat{\beta }}_{BE}$ relative to the GE loss function is given by

(25) $$\begin{array}{c} {\hat{\theta }}_{BE}={\left\{E_{\pi^{*}}{\left[\beta \right]}^{-\omega }\right\}}^{\frac{-1}{\omega }}, \end{array}$$

provided that the involved expectation *E*_*π*^∗^_[*β*]^−*ω*^ is finite. It can be shown that, when *ω* = 1, the Bayesian estimate in Eq. (25) coincides with the Bayesian estimate under the weighted squared error loss function. Similarly, when *ω* = −1, the Bayesian estimate in Eq. (25) coincides with the Bayesian estimate under the SE loss function.

By using (16), the Bayesian estimator of *λ* under GELF is given by

(26) $$\begin{array}{c} {\hat{\lambda }}_{BE}={\left\{\int_{0}^{\delta }\int_{0}^{\infty }\lambda^{-\omega }\pi^{*}\left(\lambda ,\theta \;|\;\underline{Y}\right)d\lambda d\theta \right\}}^{\frac{-1}{\omega }}={\left\{\frac{\Gamma \left(d^{*}+a_{1}-\omega \right){\left[\eta \left(\underline{y}\right)+{\tilde{R}}_{t_{1}}\ln T_{1}+\tilde{R}{}_{t_{2}}\ln T_{2}-\left(n+b_{1}\right)\ln\left(\delta \right)+\ln\left(a_{2}\right)\right]}^{\left(d^{*}+a_{1}\right)}}{\Gamma \left(d^{*}+a_{1}\right){\left[\eta \left(\underline{y}\right)+{\tilde{R}}_{t_{1}}\ln T_{1}+{\tilde{R}}_{t_{2}}\ln T_{2}-\left(n+b_{1}\right)\ln\left(\delta \right)+\ln\left(a_{2}\right)+\varepsilon \right]}^{\left(d^{*}+a_{1}-\omega \right)}}\right\}}^{\frac{-1}{\omega }} \end{array}$$

and the Bayesian estimator of *θ* under GEF is obtained as

(27) $$\begin{array}{c} {\hat{\theta }}_{BE}={\left\{\int_{0}^{\delta }\int_{0}^{\infty }\theta^{-\omega }\pi^{*}\left(\lambda ,\theta \;|\;\underline{Y}\right)d\lambda d\theta \right\}}^{\frac{-1}{\omega }}=\left\{I^{-1}\int_{0}^{\delta }\frac{\Gamma \left(d^{*}+a_{1}+1\right)}{\theta^{1-\omega }}{\left[\eta \left(\underline{y}\right)+{\tilde{R}}_{t_{1}}\ln T_{1}+{\tilde{R}}_{t_{2}}\ln T_{2}-\left(n+b_{1}\right)\ln\left(\theta \right)+\ln\left(a_{2}\right)\right]}^{\left(d^{*}+a_{1}+1\right)}d\theta \right\}. \end{array}$$

### 4.3. The Bayesian Estimation under LLF

Under the assumption that the minimal loss occurs at $\hat{\beta }=\beta$, the LINEX loss function can be expressed as

(28) $$\begin{array}{c} L_{BL}\left(\hat{\beta },\beta \right)=\exp\left[\varepsilon \left(\hat{\beta }-\beta \right)\right]-\varepsilon \left(\hat{\beta }-\beta \right)-1 \end{array}$$

where *ε* ≠ 0. The sign and magnitude of the shape parameter *v* represent the direction and degree of asymmetry, respectively. It is easily seen the (unique) Bayesian estimator of *θ*, denoted by ${\hat{\theta }}_{L}$under the LINEX loss function, and the value${\hat{\beta }}_{L}$which minimizes$E_{\pi^{*}}\left[L_{L}\left(\hat{\beta },\beta \right)\right]$is given by

(29) $$\begin{array}{c} {\hat{\beta }}_{BL}=\frac{-1}{\varepsilon }\ln\left\{E_{\pi^{*}}\left[\exp\left(-\upsilon \beta \right)\right]\right\}, \end{array}$$

provided that the involved expectation *E*_*π*^∗^_[exp(−*υβ*)] is finite.

By using (16), the Bayesian estimator of *λ* under LLF is given by

(30) $$\begin{array}{c} {\hat{\lambda }}_{BL}=\frac{-1}{\varepsilon }\ln\left\{\int_{0}^{\delta }\int_{0}^{\infty }\exp\left(-\upsilon \lambda \right)\pi^{*}\left(\lambda ,\theta \;|\;\underline{Y}\right)d\lambda d\theta \right\}=\frac{-1}{\varepsilon }\ln\left\{\frac{{\left[\eta \left(\underline{y}\right)+{\tilde{R}}_{t_{1}}\ln T_{1}+{\tilde{R}}_{t_{2}}\ln T_{2}-\left(n+b_{1}\right)\ln\left(\delta \right)+\ln\left(a_{2}\right)\right]}^{\left(d^{*}+a_{1}\right)}}{{\left[\eta \left(\underline{y}\right)+{\tilde{R}}_{t_{1}}\ln T_{1}+{\tilde{R}}_{t_{2}}\ln T_{2}-\left(n+b_{1}\right)\ln\left(\delta \right)+\ln\left(a_{2}\right)+\varepsilon \right]}^{\left(d^{*}+a_{1}\right)}}\right\}, \end{array}$$

and the Bayesian estimator of *θ* under LLF is obtained as

(31) $$\begin{array}{c} {\hat{\theta }}_{BL}=\frac{-1}{\varepsilon }\ln\left\{\int_{0}^{\delta }\int_{0}^{\infty }\exp\left(-\upsilon \theta \right)\pi^{*}\left(\lambda ,\theta \;|\;\underline{Y}\right)d\lambda d\theta \right\}=\frac{-1}{\varepsilon }\ln\left\{I^{-1}\int_{0}^{\delta }\frac{\Gamma \left(d^{*}+a_{1}+1\right)}{\theta }\exp\left(-\upsilon \theta \right)\right.\times \left.{\left[\eta \left(\underline{y}\right)+{\tilde{R}}_{t_{1}}\ln T_{1}+{\tilde{R}}_{t_{2}}\ln T_{2}-\left(n+b_{1}\right)\ln\left(\theta \right)+\ln\left(a_{2}\right)\right]}^{\left(d^{*}+a_{1}+1\right)}d\theta \right\}. \end{array}$$

## 5. One-Sample Bayesian Prediction

For $q=1,2,\cdots ,{\tilde{R}}_{j}$, let $Y_{q:{\tilde{R}}_{j}}$ denote the *q*^th^ order statistic out of ${\tilde{R}}_{j}$ removed units at stage *j*. Then, the conditional density function of $Y_{q:{\tilde{R}}_{j}}$, given the observed Type-II unified PHCS, is given, see Basak et al. [26], by

(32) $$\begin{array}{c} g\left(Y_{q:{\tilde{R}}_{j}}\;|\;\underline{Y}\right)=g\left(y\;|\;\underline{Y}\right)=\frac{{\tilde{R}}_{j}!}{\left(q-1\right)!\left({\tilde{R}}_{j}-q\right)!}\frac{{\left[G\left(y\right)-G\left(y_{j}\right)\right]}^{q-1}{\left[1-G\left(y\right)\right]}^{{\tilde{R}}_{j}-q}g\left(y\right)}{{\left[1-G\left(y_{j}\right)\right]}^{{\tilde{R}}_{j}}},\;y>y_{j}, \end{array}$$

where

(33) $$\begin{array}{c} j=\left\{\begin{array}{cc} 1,\cdots ,k,\cdots ,m-1,t_{1} & \text{in Case }1_{a},\\ 1,\cdots ,k,\cdots ,d_{1},\cdots ,m & \text{in Case }1_{b},\\ 1,\cdots ,k,\cdots ,d_{1},\cdots ,t_{2} & \text{in Cases }1_{c},\\ 1,\cdots ,d_{1},\cdots ,d_{1},\cdots ,k^{*} & \text{in Case }2_{a},\\ 1,\cdots ,d_{1},\cdots ,k,\cdots ,m & \text{in Case }2_{b},\\ 1,\cdots ,d_{1},\cdots ,k,\cdots ,t_{2} & \text{in Cases }2_{c}, \end{array}\right. \end{array}$$

with *y*_*t*_1__ = *T*_1_ and *y*_*t*_2__ = *T*_2_.

By using (6) and (7) in (32), given Type-II unified PHCS, the conditional density function of $Y_{q:{\tilde{R}}_{j}}$ is then given as follows:

(34) $$\begin{array}{c} g\left(y\;|\;\underline{Y}\right)=\overset{q-1}{\underset{h=0}{\sum }}C_{h}\frac{\lambda }{y}\exp\left\{-\lambda \left[\varpi_{h}\left(\ln y-\ln y_{j}\right)\right]\right\},y>y_{j}, \end{array}$$

where $C_{h}={\left(-1\right)}^{h}\left(\begin{array}{c} q-1\\ h \end{array}\right){\tilde{R}}_{j}!/\left(q-1\right)!\left({\tilde{R}}_{j}-q\right)!$ and $\varpi_{h}=h+{\tilde{R}}_{j}-q+1$ for *h* = 0, ⋯, *q* − 1..

Upon combining (16) and (34), the Bayesian predictive density function of $Y_{q:{\tilde{R}}_{j}}$, given UPHCS, is obtained as

(35) $$\begin{array}{c} \left(y\;|\;\underline{Y}\right)=I^{-1}\overset{q-1}{\underset{h=0}{\sum }}C_{h}\int_{0}^{\delta }\int_{0}^{\infty }\frac{\lambda^{d^{*}+a_{1}+1}}{\theta y}\exp\left\{-\lambda \left[\eta \left(\underline{y}\right)+{\tilde{R}}_{t_{1}}\ln T_{1}+{\tilde{R}}_{t_{2}}\ln T_{2}-\left(n+b_{1}\right)\ln\theta +\ln a_{2}\right]\right\}\times \exp\left\{-\lambda \left[\varpi_{h}\left(\ln y-\ln y_{j}\right)\right]\right\}d\lambda d\theta =\frac{I^{-1}\Gamma \left(d^{*}+a_{1}+1\right)}{\left(n+b_{1}\right)}\overset{q-1}{\underset{h=0}{\sum }}\frac{C_{h}}{y}{\left[\eta \left(\underline{y}\right)+{\tilde{R}}_{t_{1}}\ln T_{1}+{\tilde{R}}_{t_{2}}\ln T_{2}-\left(n+b_{1}\right)\ln\delta +\ln a_{2}+\varpi_{h}\left(\ln y-\ln y_{j}\right)\right]}^{-\left(d^{*}+a_{1}+1\right)}. \end{array}$$

The Bayesian predictive survival function of $Y_{q:{\tilde{R}}_{j}}$, given Type-II unified PHCS, is given as

(36) $$\begin{array}{c} {\bar{G}}^{*}\left(t\;|\;\underline{Y}\right)=\int_{t}^{\infty }g^{*}\left(y\;|\;\underline{Y}\right)dy=\frac{I^{-1}\Gamma \left(d^{*}+a_{1}\right)}{\left(n+b_{1}\right)}\overset{q-1}{\underset{h=0}{\sum }}\frac{C_{h}}{\varpi_{h}}{\left[\eta \left(\underline{y}\right)+{\tilde{R}}_{t_{1}}\ln T_{1}+{\tilde{R}}_{t_{2}}\ln T_{2}-\left(n+b_{1}\right)\ln\delta +\ln a_{2}+\varpi_{h}\left(\ln t-\ln y_{j}\right)\right]}^{-\left(d^{*}+a_{1}\right)}. \end{array}$$

The Bayesian point predictor of *Y* under the squared error loss function is the mean of the predictive density, given by

(37) $$\begin{array}{c} {\hat{Y}}_{q:{\tilde{R}}_{j}}=\int_{0}^{\infty }yf^{*}\left(y\;|\;\underline{Y}\right)dy, \end{array}$$

where $g^{*}\left(y|\underline{Y}\right)$ is given as in (35). The Bayesian predictive bounds of 100(1 − *α*)% two-sided equi-tailed (ET) interval for *Y*_*s*:*n*_ can be obtained by solving the following two equations:

(38) $$\begin{array}{c} {\bar{G}}^{*}\left(L_{ET}\;|\;\underline{Y}\right)=\frac{\alpha }{2}\;\text{and}\;{\bar{G}}^{*}\left(U_{ET}\;|\;\underline{Y}\right)=1-\frac{\alpha }{2}, \end{array}$$

where ${\bar{G}}^{*}\left(t|\underline{Y}\right)$ is given as in (36), and *L*_*ET*_ and *U*_*ET*_ denote the lower and upper bounds, respectively.

## 6. Two-Sample Bayesian Prediction

Let *Y*_1:*ℓ*:*m*_ ≤ *Y*_2:*ℓ*:*N*_ ≤ ⋯≤*Y*_*ℓ*:*ℓ*:*N*_ be a future independent progressive Type-II censored sample from the same population with censoring scheme $\underline{S}=\left(S_{1},\cdots ,S_{\ell }\right)$. In this section, we develop a general procedure for deriving the point and interval predictions for *Y*_*s*:*ℓ*:*N*_, 1 ≤ *s* ≤ *ℓ*, based on the observed UPHCS. The marginal density function of *Y*_*s*:*ℓ*:*N*_ is given by Balakrishnan et al. [27] as

(39) $$\begin{array}{c} g_{Y_{s:\ell :N}}\left(y_{s}\;|\;\theta \right)=C_{N,s}\overset{s-1}{\underset{h=0}{\sum }}c_{h,s-1}{\left[1-G\left(y_{s}\right)\right]}^{W_{h,s}-1}g\left(y_{s}\right), \end{array}$$

where 1 ≤ *s* ≤ *q*, *C*_*N*,*s*_ = *N*(*N* − *S*_1_ − 1) ⋯ (*N* − *S*_1_ ⋯ −*S*_*s*−1_ + 1), *W*_*h*,*s*_ = *N* − *S*_1_ − ⋯−*S*_*s*−*h*−1_ − *s* + *h* + 1, and *c*_*h*,*s*−1_ = (−1)^*h*^{[∏_*u*=1_^*h*^∑_%*ε*=*s*−*h*_^*s*−*h*+*u*−1^(*S*_*ε*_ + 1)][∏_*u*=1_^*s*−*h*−1^∑_*ε*=*u*_^*s*−*h*−1^(*S*_*ε*_ + 1)]}^−1^..

Upon substituting (7) and (6) in (39), the marginal density function of *Y*_*s*:*ℓ*:*N*_ is then obtained as

(40) $$\begin{array}{c} g_{Y_{s:\ell :N}}\left(y_{s}\;|\;\theta \right)=C_{N,s}\overset{s-1}{\underset{h=0}{\sum }}c_{h,s-1}\frac{\lambda }{y_{s}}\exp\left\{-\lambda \left[W_{h,s}\ln\left(\frac{y_{s}}{\%\theta }\right)\right]\right\},\\ y_{s}>0. \end{array}$$

Upon combining (16) and (39), given UPHCS, the Bayesian predictive density function of *Y*_*s*:*ℓ*:*N*_ is obtained as

(41) $$\begin{array}{c} g_{Y_{s:\ell :N}}^{*}\left(y_{s}\;|\;\underline{Y}\right)=\left\{\begin{array}{cc} g_{1Y_{s:\ell :N}}^{*}\left(y_{s}\;|\;\underline{Y}\right), & 0<y_{s}\leq \delta ,\\ g_{2Y_{s:\ell :N}}^{*}\left(y_{s}\;|\;\underline{Y}\right), & y_{s}>\delta , \end{array}\right. \end{array}$$

where

(42) $$\begin{array}{c} g_{1Y_{s:\ell :N}}^{*}\left(y_{s}\;|\;\underline{Y}\right)=\int_{0}^{y_{s}}\int_{0}^{\infty }g_{Y_{s:\ell :N}}\left(y_{s}\;|\;\underline{Y}\right)\pi^{*}\left(\lambda ,\theta \;|\;\underline{Y}\right)d\lambda d\theta =I^{-1}\Gamma \left(d^{*}+a_{1}+1\right)C_{N,s}\overset{s-1}{\underset{h=0}{\sum }}\frac{c_{h,s-1}}{\%\left(n+b_{1}+W_{h,s}\right)y_{s}}\times {\left[\eta \left(\underline{y}\right)+{\tilde{R}}_{t_{1}}\ln T_{1}+{\tilde{R}}_{t_{2}}\ln T_{2}-\left(n+b_{1}\right)\ln y_{s}+\ln a_{2}\right]}^{-\left(d^{*}+a_{1}+1\right)},\\ g_{2Y_{s:\ell :N}}^{*}\left(y_{s}\;|\;\underline{Y}\right)=\int_{0}^{\delta }\int_{0}^{\infty }g_{Y_{s:\ell :N}}\left(y_{s}\;|\;\underline{Y}\right)\pi^{*}\left(\lambda ,\theta \;|\;\underline{Y}\right)d\lambda d\theta =I^{-1}\Gamma \left(d^{*}+a_{1}+1\right)C_{N,s}\overset{q-1}{\underset{h=0}{\sum }}\frac{c_{h,s-1}}{\left(n+b_{1}+W_{h,s}\right)y_{s}}\times {\left[\eta \left(\underline{y}\right)+{\tilde{R}}_{t_{1}}\ln T_{1}+{\tilde{R}}_{t_{2}}\ln T_{2}-\left(n+b_{1}+W_{h,s}\right)\ln\delta +W_{h,s}\ln y_{s}+\ln a_{2}\right]}^{-\left(d^{*}+a_{1}+1\right)}. \end{array}$$

From (41), we simply obtain the predictive survival function of *Y*_*s*:*ℓ*:*N*_, given UPHCS, as

(43) $$\begin{array}{c} {\bar{G}}_{Y_{s:\ell :N}}^{*}\left(t\;|\;\underline{Y}\right)=\int_{t}^{\infty }g^{*}\left(y_{s}\;|\;\underline{Y}\right){dy}_{s}=\left\{\begin{array}{cc} {\bar{G}}_{1Y_{s:\ell :N}}^{*}\left(t\;|\;\underline{Y}\right), & 0<t\leq \delta ,\\ {\bar{G}}_{2Y_{s:\ell :N}}^{*}\left(t\;|\;\underline{Y}\right), & t>\delta , \end{array}\right. \end{array}$$

where

(44) $$\begin{array}{c} {\bar{G}}_{1Y_{s:\ell :N}}^{*}\left(t\;|\;\underline{Y}\right)=\int_{0_{t}}^{\delta_{\infty }}g_{1Y_{s:\ell :N}}^{*}\left(y_{s}\;|\;\underline{Y}\right){dy}_{s}+\int_{0_{\delta }}^{\infty_{\infty }}g_{2Y_{s:\ell :N}}^{*}\left(y_{s}\;|\;\underline{Y}\right){dy}_{s}=I^{-1}\Gamma \left(d^{*}+a_{1}\right)C_{N,s}\overset{s-1}{\underset{h=0}{\sum }}\frac{c_{h,s-1}}{\left(n+b_{1}\right)\left(n+b_{1}+W_{h,s}\right)W_{h,s}}\times \left\{\left(n+b_{1}+W_{h,s}\right){\left[\eta \left(\underline{y}\right)+{\tilde{R}}_{t_{1}}\ln T_{1}+{\tilde{R}}_{t_{2}}\ln T_{2}-\left(n+b_{1}\right)\ln\delta +\ln a_{2}\right]}^{-\left(d^{*}+a_{1}\right)}\right.-\left.W_{h,s}{\left[\eta \left(\underline{y}\right)+{\tilde{R}}_{t_{1}}\ln T_{1}+{\tilde{R}}_{t_{2}}\ln T_{2}-\left(n+b_{1}\right)\ln t+\ln a_{2}\right]}^{-\left(d^{*}+a_{1}\right)}\right\}\\ {\bar{G}}_{2Y_{s:\ell :N}}^{*}\left(t\;|\;\underline{Y}\right)=\int_{0_{t}}^{\infty_{\infty }}g_{2Y_{s:\ell :N}}^{*}\left(y_{s}\;|\;\underline{Y}\right){dy}_{s}=I^{-1}\Gamma \left(d^{*}+a_{1}\right)C_{N,s}\overset{s-1}{\underset{h=0}{\sum }}\frac{c_{h,s-1}}{W_{h,s}\left(n+b_{1}+W_{h,s}\right)}\times {\left[\eta \left(\underline{y}\right)+{\tilde{R}}_{t_{1}}\ln T_{1}+{\tilde{R}}_{t_{2}}\ln T_{2}-\left(n+b_{1}+W_{h,s}\right)\ln\delta +W_{h,s}\ln t+\ln a_{2}\right]}^{-\left(d^{*}+a_{1}\right)}. \end{array}$$

The Bayesian point predictor of *Y*_*s*:*ℓ*:*N*_, 1 ≤ *s* ≤ *m*, under the squared error loss function is the mean of the predictive density, given by

(45) $$\begin{array}{c} {\hat{Y}}_{s:\ell :N}=\int_{0}^{\infty }y_{s}g_{Y_{s\ell :N}}^{*}\left(y_{s}\;|\;\underline{Y}\right){dy}_{s}, \end{array}$$

where $g_{Y_{s:\ell :N}}^{*}\left(y_{s}|\underline{Y}\right)$ is given as in (41).

The Bayesian predictive bounds of 100(1 − *α*)% ET interval for *Y*_*s*:*ℓ*:*N*_, 1 ≤ *s* ≤ *m*, can be obtained by solving the following two equations:

(46) $$\begin{array}{c} {\bar{G}}_{Y_{s:\ell :N}}^{*}\left(L_{ET}\;|\;\underline{Y}\right)=\frac{\alpha }{2}\text{ and }{\bar{G}}_{Y_{s:\ell :N}}^{*}\left(U_{ET}\;|\;\underline{Y}\right)=1-\frac{\alpha }{2}, \end{array}$$

where ${\bar{G}}_{Y_{s:\ell :N}}^{*}\left(t|\underline{Y}\right)$ is given as in (43), and *L*_*ET*_ and *U*_*ET*_ denote the lower and upper bounds, respectively.

## 7. Simulation Study

In this section, we present a simulation study to compare the performance of the classical ML and Bayesian estimation procedures under different Type-II unified PHCS. Extensive computations were performed using the statistical software maple.

Firstly, we show how we generate Type-II unified PHC data from Pareto distribution. For given values of *n*, *m*, *T*_1_, *T*_2_, and *R* = (*R*_1_, ⋯, *R*_*m*_). We will use the transformation which was suggested by Balakrishnan and Aggarwala in [28] to generate Type-II progressive censored data from Pareto distribution. Let the generated Type-II PC data is (*y*_1,*m*,*n*_, *y*_2,*m*,*n*_, ⋯, *y*_*m*,*m*,*n*_), if *y*_*m*,*mn*_ < *T*_1_, we set *R*_*m*_ = 0 and use the transformation which was suggested by Ng et al. in [29] to generate *R*_*m*_ order statistics from left truncated Pareto distribution with truncated value *y*_*m*,*m*,*n*_. Now, we *m* Type-II progressive censored data and *R*_*m*_ order statistics as the following (*y*_1,*m*,*n*_, *y*_2,*m*,*n*_, ⋯, *y*_*m*,*m*,*n*_, *y*_*m*+1,*n*_, *y*_*m*+*R*_*m*_,*n*_). Then, we determined the termination time of the experiment and the corresponding observed Type-II unified PHC data as shown in Section 2.

We simulate Type-II unified PHCS for different combinations for a sample of size *n* = 50, with different values of *m* = 2*k*, and *T*_2_ = 2*T*_1_ from the Pareto distribution. For convenience, we consider the true values of the unknown parameters as *λ* = 1 and *θ* = 3.

For the point estimate, we computed the ML estimate and Bayesian estimates of *λ* and *θ,* under SELF, LLF (with *ε* = 0.5), and GELF (with *ω* = 0.5) using informative prior (IP) and non-informative priors (NIP) values for the mean square error (MSE) and the estimated bias (EB) for each estimate. We construct also the average confidence length (ACL) and the coverage probabilities (CP) of the 90% and 95% asymptotic confidence intervals and Bayesian credible intervals for *λ*_b_ and *θ*_b_, using 1,000 simulations.

We take the different censoring schemes as follows:

1. Scheme 1 *R*_*m*_ = *R*_*k*_ = *n* − *m*/2, *R*_*i*_ = 0 for all *i*≠*k*, *m*.
2. Scheme 2 *R*_1_ = *R*_*m*_ = *n* − *m*/2, *R*_*i*_ = 0 for all *i*≠1, *m*..

The average estimates, MSE and EB for ML and Bayesian estimates of *λ* and *θ*, have been reported in Tables 1 and 2, respectively, also, Tables 3 and 4 are present the ACL of 90% and 95% confidence intervals with corresponding CP for $\hat{\lambda }$ and $\hat{\theta }$, respectively.

## 8. Numerical Example

In this section, we use the real data set to show the performance of the inferential results established for the Pareto distribution based on the Type-II unified PHSC, in addition to comparing ML and Bayesian estimates through Monte Carlo simulations. This real data set contains the failure times (in hours) of one plane's ac system from a pair of real data sets collected by Bain and Engelhardt [30]. Moreover, Guo and Gui [31] demonstrated that these data sets closely matched the inverse Pareto distribution. For further proceeding, before using these data, we ran Kolmogorov-Smirnov (KS) goodness of fit tests to see if they followed the Pareto distribution or not. For these data sets, the KS test statistics with their related *p*-values are more than 0.05, so we can assume that these data sets follow Pareto distribution at a 0.05% level of significance. This real data are ordered in Table 5.

We will use these data to generate the Type-II unified PHCS, suppose *m* = 9, *k* = 6, *R*_*i*_ = 2 for *i* = 3,6,9, and *R*_*i*_ = 0 otherwise with different values of *T*_1_ and *T*_2_ with *T*_2_ = 2 *T*_1_.  Table 6 shows different Type-II unified PHCSs.

After generating the Type-II unified PHC data with the different unified PHCS, we ran KS goodness of fit tests for all Type-II unified PHC data to see if they followed the Pareto distribution or not. For all these Type-II unified PHC data sets, the KS test statistics with their related *p*-values are more than 0.05, so we can assume that these data and all generated Type-II unified PHC data sets from it follow Pareto distribution at a 0.05% level of significance.

Based on the Type-II unified PHCS and two different choices IP and NIP priors, the ML and Bayesian estimates for the unknown parameters *λ* and *θ* are presented in Tables 7 and 8. Moreover, the 95% and 99% asymptotic confidence intervals and the credible intervals are presented in Tables 9 and 10. Finally, Tables 11 and 12 present the point predictor with 95% and 99% Bayesian prediction bounds of *Y*_*s*:*ℓ*:*N*_ from the future progressively censored sample of size *ℓ* = 10 from a sample of size *N* = 20 with progressive censoring scheme *S* = (0,2,0,2,0,2,0,2,0,2) for four different choices of censoring schemes.

Since *R*_1_ = 0, then *y*_1_ = 1.2 is not removed from censored data in all Type-II unified PHCS, and since ${\hat{\theta }}_{ML}=y_{1}$ so that ${\hat{\theta }}_{ML}=1.2$ in all four Type-II unified PHCS.

## 9. Conclusions and Discussion

From Tables 1 and 2, we observe that the MSEs of the Bayesian estimates based on the LINEX, GE, and SE loss functions are smaller than those of the ML estimates. Furthermore, the MSEs and EBs of all estimates decrease with increasing *m* and *k* when *T*_1_ and *T*_2_ are fixed. Also, the MSEs and EBs of all estimates decrease with increasing *T*_1_ and *T*_2_ when *m* and *k* are fixed. Moreover, a comparison of the results for the informative priors with the corresponding ones for non-informative priors reveals that the former produces more precise results.

From the results in Tables 10 and 11, we notice that the point predictor of mean is between the upper and lower bounds of the prediction intervals. Additionally, as we would expect, a comparison of the results for the informative prior with the corresponding ones for non-informative prior reveals that the former produces more precise results, because the interval length in the informative prior case is short than in non-informative case. Moreover, the 95% prediction intervals seem to be more precise than the 99% prediction intervals, Finally when we use the same value of *T*_1_ and *T*_2_ but increasing *k* and *m*. , the Bayesian prediction bounds become tighter as expected since the duration of the life-testing experiment is longer in this case.

## Figures and Tables

**Table 1:** The values of MSE and EB of ML and Bayesian estimates for *λ* based on the different Type-II unified PHCSs.

(*n*, *m*, *k*)	Sch.	(*T*_1_, *T*_2_)	${\hat{\lambda }}_{ML}$	${\hat{\lambda }}_{B}$					
				${\hat{\lambda }}_{BS}$		${\hat{\lambda }}_{BE}$		${\hat{\lambda }}_{BL}$	
				IP	NIP	IP	NIP	IP	NIP
			*MSE*						
(50,20,10)	1	(5,10)	0.2637	0.2075	0.2341	0.1954	0.2191	0.1999	0.2247
	2		0.2823	0.2215	0.2516	0.2083	0.2353	0.2133	0.2414
(50,30,15)	1		0.2192	0.1891	0.2053	0.1837	0.1989	0.1851	0.2006
	2		0.2193	0.1899	0.2064	0.1854	0.2010	0.1861	0.2020
(50,40,20)	1		0.2009	0.1794	0.1920	0.1768	0.1889	0.1768	0.1890
	2		0.1996	0.1782	0.1904	0.1751	0.1869	0.1755	0.1873
(50,20,10)	1	(10,20)	0.2382	0.1868	0.2107	0.1759	0.1972	0.1799	0.2022
	2		0.1949	0.2158	0.2333	0.1875	0.2118	0.1920	0.2406
(50,30,15)	1		0.1503	0.1331	0.1420	0.1326	0.1412	0.1314	0.1400
	2		0.1672	0.1452	0.1555	0.1419	0.1516	0.1425	0.1523
(50,40,20)	1		0.1672	0.1452	0.1555	0.1419	0.1516	0.1425	0.1523
	2		0.1877	0.1676	0.1779	0.1633	0.1732	0.1647	0.1747
(50,20,10)	1	(15,30)	0.2144	0.2300	0.2474	0.2531	0.2724	0.2356	0.2534
	2		0.1754	0.1942	0.2100	0.2186	0.2363	0.2005	0.2165
(50,30,15)	1		0.1208	0.1320	0.1396	0.1193	0.1271	0.1183	0.1260
	2		0.1098	0.1173	0.1241	0.1311	0.1387	0.1208	0.1278
(50,40,20)	1		0.1505	0.1307	0.1400	0.1277	0.1364	0.1283	0.1371
	2		0.1770	0.1581	0.1674	0.1539	0.1627	0.1554	0.1643

			*EB*						
(50,20,10)	1	(5,10)	0.1102	0.0459	0.0547	0.0086	0.0131	0.0326	0.0397
	2		0.1178	0.0516	0.0618	0.0141	0.0199	0.0382	0.0465
(50,30,15)	1		0.0669	0.0265	0.0299	0.0006	0.0021	0.0175	0.0202
	2		0.0642	0.0232	0.0261	0.0033	0.0024	0.0140	0.0162
(50,40,20)	1		0.0515	0.0167	0.0184	0.0065	0.0064	0.0088	0.0099
	2		0.0527	0.0187	0.0205	0.0039	0.0036	0.0110	0.0122
(50,20,10)	1	(10,20)	0.0992	0.0413	0.0492	0.0077	0.0118	0.0293	0.0357
	2		0.1060	0.0464	0.0556	0.0127	0.0179	0.0344	0.0419
(50,30,15)	1		0.0319	0.0030	0.0025	0.0005	0.0019	0.0111	0.0111
	2		0.0480	0.0113	0.0130	0.0030	0.0022	0.0030	0.0041
(50,40,20)	1		0.0464	0.0150	0.0166	0.0051	0.0061	0.0079	0.0089
	2		0.0474	0.0168	0.0185	0.0035	0.0032	0.0099	0.0110
(50,20,10)	1	(15,30)	0.2071	0.2243	0.2417	0.2484	0.2677	0.2303	0.2480
	2		0.1674	0.1884	0.2040	0.2138	0.2314	0.1950	0.2111
(50,30,15)	1		0.0287	0.0027	0.0023	0.0244	0.0254	0.0100	0.0100
	2		0.0470	0.0102	0.0117	0.0119	0.0119	0.0027	0.0037
(50,40,20)	1		0.0520	0.0233	0.0254	0.0044	0.0054	0.0168	0.0184
	2		0.0510	0.0225	0.0245	0.0036	0.0046	0.0160	0.0176

**Table 2:** The values of MSE and EB of ML and Bayesian estimates for *θ* based on the different Type-II unified UHCSs.

(*n*, *m*, *k*)	Sch.	(*T*_1_, *T*_2_)	${\hat{\theta }}_{ML}$	${\hat{\theta }}_{B}$					
				${\hat{\theta }}_{BS}$		${\hat{\theta }}_{BE}$		${\hat{\theta }}_{BL}$	
				IP	NIP	IP	NIP	IP	NIP
			*MSE*						
(50,20,10)	1	(5,10)	0.0820	0.0604	0.0673	0.0671	0.0674	0.0544	0.0598
	2		0.0911	0.0671	0.0674	0.0672	0.0675	0.0604	0.0664
(50,30,15)	1		0.0771	0.0569	0.0634	0.0570	0.0572	0.0512	0.0563
	2		0.0857	0.0632	0.0635	0.0633	0.0636	0.0569	0.0626
(50,40,20)	1		0.0758	0.0602	0.0604	0.0603	0.0605	0.0542	0.0596
	2		0.0842	0.0601	0.0603	0.0602	0.0604	0.0541	0.0595
(50,20,10)	1	(10,20)	0.0738	0.0544	0.0606	0.0604	0.0607	0.0489	0.0538
	2		0.0820	0.0604	0.0607	0.0605	0.0608	0.0544	0.0598
(50,30,15)	1		0.0694	0.0512	0.0631	0.0513	0.0515	0.0461	0.0507
	2		0.0771	0.0630	0.0631	0.0631	0.0633	0.0567	0.0623
(50,40,20)	1		0.0682	0.0600	0.0601	0.0601	0.0602	0.0540	0.0594
	2		0.0758	0.0600	0.0601	0.0600	0.0602	0.0540	0.0594
(50,20,10)	1	(15,30)	0.0664	0.0489	0.0545	0.0544	0.0546	0.0440	0.0484
	2		0.0738	0.0544	0.0546	0.0544	0.0547	0.0489	0.0538
(50,30,15)	1		0.0625	0.0461	0.0568	0.0461	0.0464	0.0415	0.0456
	2		0.0694	0.0567	0.0568	0.0568	0.0570	0.0510	0.0561
(50,40,20)	1		0.0614	0.0540	0.0541	0.0600	0.0542	0.0486	0.0535
	2		0.0682	0.0599	0.0600	0.0540	0.0601	0.0486	0.0593

			EB						
(50,20,10)	1	(5,10)	0.0555	0.0005	0.0010	0.0006	0.0021	0.0004	0.0005
	2		0.0617	0.0006	0.0009	0.0005	0.0020	0.0005	0.0006
(50,30,15)	1		0.0519	0.0034	0.0048	0.0045	0.0059	0.0031	0.0034
	2		0.0577	0.0037	0.0052	0.0048	0.0063	0.0034	0.0037
(50,40,20)	1		0.0526	0.0031	0.0045	0.0041	0.0056	0.0028	0.0030
	2		0.0584	0.0029	0.0043	0.0039	0.0053	0.0026	0.0028
(50,20,10)	1	(10,20)	0.0500	0.0005	0.0009	0.0005	0.0019	0.0004	0.0005
	2		0.0555	0.0005	0.0008	0.0005	0.0018	0.0005	0.0005
(50,30,15)	1		0.0467	0.0031	0.0043	0.0041	0.0053	0.0028	0.0031
	2		0.0519	0.0036	0.0049	0.0046	0.0060	0.0032	0.0035
(50,40,20)	1		0.0473	0.0020	0.0033	0.0030	0.0043	0.0018	0.0020
	2		0.0526	0.0019	0.0032	0.0029	0.0042	0.0017	0.0019
(50,20,10)	1	(15,30)	0.0450	0.0004	0.0008	0.0005	0.0017	0.0003	0.0004
	2		0.0500	0.0005	0.0007	0.0004	0.0016	0.0004	0.0005
(50,30,15)	1		0.0421	0.0028	0.0039	0.0036	0.0048	0.0025	0.0028
	2		0.0467	0.0032	0.0044	0.0041	0.0054	0.0029	0.0032
(50,40,20)	1		0.0426	0.0019	0.0031	0.0029	0.0041	0.0017	0.0019
	2		0.0473	0.0017	0.0031	0.0026	0.0038	0.0015	0.0017

**Table 3:** The ACL of 95% and 99% confidence intervals and corresponding CP for ${\hat{\lambda }}_{ML}$ and ${\hat{\lambda }}_{B}$ at the different priors and Type-II unified PHCSs.

(*n*, *m*, *k*)	Sch.	95%							99%					
		${\hat{\lambda }}_{ML}$			${\hat{\lambda }}_{B}$				${\hat{\lambda }}_{ML}$		${\hat{\lambda }}_{B}$			
					IP		NIP				IP		NIP	
		(*T*_1_, *T*_2_)	ACL	CP	ACL	CP	ACL	CP	ACL	CP	ACL	CP	ACL	CP
(50,20,10)	1	(5,10)	0.988	0.985	0.940	0.979	0.968	0.996	1.391	0.990	1.240	0.979	1.257	1.000
	2		0.988	0.977	0.940	0.971	0.968	0.993	1.391	0.986	1.240	0.977	1.253	0.989
(50,30,15)	1		0.800	0.981	0.761	0.973	0.786	0.981	1.134	0.991	1.003	0.988	1.089	0.983
	2		0.682	0.985	0.650	0.981	0.654	0.997	0.924	0.986	0.820	0.982	0.869	0.975
(50,40,20)	1		0.532	1.000	0.506	0.979	0.513	0.978	0.758	0.995	0.672	1.000	0.716	0.989
	2		0.410	0.986	0.384	0.977	0.509	1.000	0.752	1.000	0.667	1.000	0.711	1.000
(50,20,10)	1	(10,20)	0.677	0.991	0.643	0.988	0.675	0.995	0.954	0.976	0.849	0.980	0.875	0.985
	2		0.711	0.986	0.675	0.982	0.707	0.989	1.001	0.977	0.891	1.000	0.917	0.978
(50,30,15)	1		0.789	0.995	0.750	1.000	0.775	0.983	1.109	0.984	0.989	0.974	1.004	0.989
	2		0.800	1.000	0.761	1.000	0.786	0.975	1.125	0.986	1.003	0.982	1.018	0.984
(50,40,20)	1		0.601	0.976	0.572	0.980	0.583	0.989	0.813	0.984	0.726	0.979	0.727	0.990
	2		0.793	0.977	0.754	0.997	0.777	0.972	1.114	1.000	0.993	0.974	1.006	1.000
(50,20,10)	1	(15,30)	0.541	0.984	0.514	0.974	0.544	0.985	0.764	0.983	0.678	0.974	0.710	0.971
	2		0.563	0.986	0.534	0.982	0.564	0.978	0.794	0.991	0.705	0.987	0.737	0.994
(50,30,15)	1		0.681	0.984	0.648	0.979	0.673	0.989	0.938	1.000	0.854	0.988	0.703	1.000
	2		0.702	1.000	0.667	0.974	0.692	0.984	0.969	0.978	0.879	0.986	0.751	0.995
(50,40,20)	1		0.793	0.983	0.754	0.974	0.777	0.990	1.114	0.992	0.993	0.992	1.003	0.984
	2		0.793	0.991	0.754	0.987	0.777	1.000	1.117	0.975	0.993	1.000	1.032	0.986

**Table 4:** The ACL of 95% and 99% confidence intervals and corresponding CP for ${\hat{\theta }}_{ML}$ and ${\hat{\theta }}_{B}$ at the different priors and Type-II unified PHCSs.

(*n*, *m*, *k*)	Sch.	95%							99%					
		${\hat{\theta }}_{ML}$			${\hat{\theta }}_{B}$						${\hat{\theta }}_{B}$			
					IP		NIP		${\hat{\theta }}_{ML}$		IP		NIP	
		(*T*_1_, *T*_2_)	ACL	CP	ACL	CP	ACL	CP	ACL	CP	ACL	CP	ACL	CP
(50,20,10)	1	(5,10)	0.269	0.963	0.249	0.943	0.263	0.945	0.405	0.992	0.354	0.990	0.375	0.990
	2		0.370	0.963	0.351	0.944	0.354	0.945	0.512	0.991	0.456	0.990	0.466	0.989
(50,30,15)	1		2.447	0.969	2.379	0.950	2.282	0.950	2.699	0.983	2.478	0.983	2.385	0.980
	2		2.757	0.953	2.749	0.945	2.503	0.923	3.019	0.965	2.845	0.976	2.595	0.951
(50,40,20)	1		4.188	0.973	4.073	0.955	3.904	0.953	4.536	0.982	4.170	0.982	4.004	0.978
	2		4.276	0.978	4.151	0.957	3.994	0.960	4.629	0.984	4.246	0.984	4.093	0.980
(50,20,10)	1	(10,20)	0.326	0.986	0.298	0.965	0.322	0.968	0.505	0.995	0.437	0.993	0.473	0.993
	2		0.309	0.982	0.283	0.962	0.305	0.964	0.480	0.995	0.416	0.994	0.449	0.993
(50,30,15)	1		0.294	0.964	0.276	0.942	0.285	0.948	0.428	0.988	0.378	0.986	0.392	0.987
	2		0.437	0.962	0.414	0.942	0.418	0.945	0.577	0.988	0.515	0.986	0.525	0.987
(50,40,20)	1		4.574	0.984	4.469	0.963	4.244	0.966	4.944	0.993	4.565	0.991	4.344	0.991
	2		4.564	0.987	4.523	0.966	4.169	0.969	4.933	0.996	4.619	0.994	4.269	0.994
(50,20,10)	1	(15,30)	0.395	0.983	0.361	0.965	0.392	0.963	0.609	0.995	0.526	0.994	0.572	0.993
	2		0.378	0.985	0.346	0.967	0.375	0.965	0.584	0.995	0.504	0.993	0.548	0.994
(50,30,15)	1		0.280	0.968	0.261	0.948	0.273	0.950	0.423	0.990	0.372	0.988	0.390	0.988
	2		0.287	0.967	0.268	0.949	0.279	0.948	0.427	0.990	0.377	0.989	0.393	0.988
(50,40,20)	1		2.774	0.976	2.940	0.956	2.343	0.957	3.041	0.991	3.037	0.989	2.443	0.990
	2		2.402	0.973	2.644	0.953	1.931	0.955	2.648	0.991	2.741	0.989	2.031	0.990

**Table 5:** The real data.

1.2	2.1	2.6	2.7	2.9	2.9	4.8	5.7	5.9	7.0	7.4	15.3	32.6	38.6	50.2

**Table 6:** The different Type-II unified HPCS with (*m*, *k*) = (9, 6) and different choices of *T*_1_ and *T*_2_.

*Scheme*1	(*t*_1_, *t*_2_) = (2, 4)
	*T* ^∗^ = *X*_*k*:*m*:*n*_
	*d* ^∗^ = 6
	$\underline{Y}=\left(1.2,2.1,2.6,2.7,2.9,4.8\right)$
	$\tilde{R}=\left(0,0,2,0,0,7\right)$
	$\left({\tilde{R}}_{t_{1}},{\tilde{R}}_{t_{2}}\right)=\left(0,0\right)$
*Scheme*2	(*t*_1_, *t*_2_) = (3, 6)
	*T* ^∗^ = *t*_2_
	*d* ^∗^ = 7
	$\underline{Y}=\left(1.2,2.1,2.6,2.7,2.9,4.8,5.7\right)$
	$\tilde{R}=\left(0,0,2,0,0,2,0\right)$
	$\left({\tilde{R}}_{t_{1}},{\tilde{R}}_{t_{2}}\right)=\left(0,4\right)$
*Scheme*3	(*t*_1_, *t*_2_) = (6, 12)
	*T* ^∗^ = *X*_*m*:*m*:*n*_
	*d* ^∗^ = 9
	$\underline{Y}=\left(1.2,2.1,2.6,2.7,2.9,4.8,5.7,7.0,7.4\right)$
	$\tilde{R}=\left(0,0,2,0,0,2,0,0,2\right)$
	$\left({\tilde{R}}_{t_{1}},{\tilde{R}}_{t_{2}}\right)=\left(0,0\right)$
*Scheme*4	(*t*_1_, *t*_2_) = (10, 20)
	*T* ^∗^ = *t*_1_
	*d* ^∗^ = 9
	$\underline{Y}=\left(1.2,2.1,2.6,2.7,2.9,4.8,5.7,7.0,7.4\right)$
	$\tilde{R}=\left(0,0,2,0,0,2,0,0,0\right)$
	$\left({\tilde{R}}_{t_{1}},{\tilde{R}}_{t_{2}}\right)=\left(2,0\right)$

**Table 7:** The ML and Bayesian estimates of *λ* based on the different Type-II unified PHCSs from real data.

Sch.	${\hat{\lambda }}_{ML}$	${\hat{\lambda }}_{B}$					
		${\hat{\lambda }}_{BS}$		${\hat{\lambda }}_{BE}$		${\hat{\lambda }}_{BL}$	
		IP	NIP	IP	NIP	IP	NIP
1	0.3831	0.3504	0.3192	0.3108	0.2718	0.3458	0.3142
2	0.4320	0.3964	0.3780	0.3620	0.3378	0.3919	0.3730
3	0.5140	0.4641	0.4569	0.4280	0.4143	0.4586	0.4505
4	0.4898	0.4493	0.4408	0.4177	0.4043	0.4446	0.4355

**Table 8:** The 95% and 99% confidence intervals estimates of *λ* based on the different Type-II unified PHCSs from real data.

Sch.	95%						99%					
	${\hat{\lambda }}_{ML}$		${\hat{\lambda }}_{B}$						${\hat{\lambda }}_{B}$			
			IP		NIP		${\hat{\lambda }}_{ML}$		IP		NIP	
	LB	UB	LB	UB	LB	UB	LB	UB	LB	UB		UB
1	0.2494	0.7597	0.1362	0.6639	0.1037	0.6539	0.1474	0.8618	0.0973	0.7995	0.0688	0.8041
2	0.3453	0.9182	0.1774	0.7020	0.1520	0.7052	0.2308	1.0328	0.1339	0.8299	0.1100	0.8456
3	0.3453	0.9182	0.2186	0.8005	0.1972	0.8237	0.2308	1.0328	0.1683	0.9395	0.1468	0.9785
4	0.3113	0.7802	0.2209	0.7575	0.2016	0.7721	0.2175	0.8740	0.1728	0.8834	0.1534	0.9100

**Table 9:** The ML and Bayesian estimates of *θ* based on the different Type-II unified PHCSs from real data.

Sch.	${\hat{\theta }}_{ML}$	${\hat{\theta }}_{B}$					
		${\hat{\theta }}_{BS}$		${\hat{\theta }}_{BE}$		${\hat{\theta }}_{BL}$	
		IP	NIP	IP	NIP	IP	NIP
1	1.2000	1.0093	0.9623	0.9092	0.8674	1.0009	0.9499
2	1.2000	1.0093	0.9623	0.9092	0.8674	1.0009	0.9499
3	1.2000	1.0551	1.0317	0.9501	0.9292	1.0501	1.0251
4	1.2000	1.0522	1.0284	0.9475	0.9262	1.0471	1.0217

**Table 10:** The 95% and 99% confidence intervals estimates of *θ* based on the different Type-II unified PHCSs from real data.

Sch.	95%						99%					
	${\hat{\theta }}_{ML}$		${\hat{\theta }}_{B}$				${\hat{\theta }}_{ML}$		${\hat{\theta }}_{B}$			
			IP		NIP				IP		NIP	
	LB	UB	LB	UB	LB	UB	LB	UB	LB	UB	LB	UB
1	0.4985	1.3143	0.5297	1.1950	0.3840	1.1937	0.3126	1.3189	0.3126	1.1990	0.1676	1.1987
2	0.4985	1.3143	0.5297	1.1950	0.3840	1.1937	0.3126	1.3189	0.3126	1.1990	0.1676	1.1987
3	0.6346	1.3158	0.6842	1.1962	0.6056	1.1956	0.4961	1.3192	0.4961	1.1992	0.4009	1.1991
4	0.6297	1.3156	0.6792	1.1961	0.6022	1.1954	0.4944	1.3191	0.4944	1.1992	0.4030	1.1991

**Table 11:** Bayesian point predictor with 95% and 99% ET prediction intervals for $Y_{q:{\tilde{R}}_{j}}$ for $q=1,\cdots ,{\tilde{R}}_{j}$, with *j* = 1, ⋯, *d*^∗^, ${\tilde{R}}_{t_{1}}$, and ${\tilde{R}}_{t_{2}}$.

Sch.	*j*	*q*	95%					99%				
			${\hat{X}}_{q:R_{j}^{*}}$	IP		NIP		${\hat{X}}_{q:R_{j}^{*}}$	IP		NIP	
				LB	UB	LB	UB		LB	UB	LB	UB
1	3	1	5.22	1.883	8.561	1.695	9.417	7.830	3.305	12.354	2.975	13.590
		2	7.61	4.271	10.948	3.843	12.043	10.217	5.692	14.741	5.123	16.215
	6	1	8.33	4.993	11.671	4.494	12.838	10.939	6.415	15.464	5.773	17.010
		2	12.19	8.851	15.529	7.966	17.082	14.798	10.273	19.322	9.246	21.255
		3	18.09	14.750	21.427	13.275	23.570	20.696	16.172	25.221	14.555	27.743
		4	22.24	18.903	25.581	17.013	28.139	24.849	20.325	29.374	18.292	32.311
		5	26.79	23.449	30.127	21.104	33.139	29.396	24.871	33.920	22.384	37.312
		6	33.63	30.295	36.972	27.265	40.669	36.241	31.716	40.765	28.545	44.842
		7	62.51	59.169	65.847	53.252	72.431	65.116	60.591	69.640	54.532	76.604

2	3	1	7.39	4.046	10.724	3.642	11.796	9.993	5.468	14.517	4.921	15.969
		2	10.90	7.557	14.234	6.801	15.658	13.503	8.979	18.028	8.081	19.830
	6	1	12.58	9.242	15.920	8.318	17.512	15.189	10.664	19.713	9.598	21.684
		2	18.88	15.546	22.224	13.992	24.446	21.493	16.968	26.017	15.271	28.619
	*t*_2_	1	11.78	8.444	15.122	7.600	16.634	14.391	9.866	18.915	8.880	20.807
		2	17.16	13.822	20.499	12.440	22.549	19.768	15.244	24.293	13.719	26.722
		3	23.07	19.726	26.404	17.754	29.044	25.673	21.148	30.197	19.033	33.217
		4	30.68	27.337	34.014	24.603	37.416	33.283	28.759	37.808	25.883	41.589

3	3	1	9.04	5.706	12.384	5.136	13.622	11.653	7.128	16.177	6.415	17.795
		2	14.43	11.093	17.770	9.983	19.547	17.039	12.514	21.563	11.263	23.720
	6	1	10.44	7.105	13.783	6.395	15.161	13.052	8.527	17.576	7.675	19.334
		2	15.41	12.070	18.747	10.863	20.622	18.016	13.492	22.541	12.142	24.795
	9	1	16.66	13.325	20.002	11.993	22.003	19.271	14.747	23.796	13.272	26.175
		2	26.15	22.815	29.492	20.533	32.441	28.761	24.236	33.286	21.813	36.614

4	3	1	23.13	19.791	26.468	17.811	29.115	25.737	21.212	30.261	19.091	33.287
		2	38.14	34.798	41.475	31.318	45.623	40.744	36.220	45.269	32.598	49.796
	6	1	17.79	14.453	21.131	13.008	23.244	20.400	15.875	24.924	14.288	27.417
		2	26.71	23.369	30.046	21.032	33.051	29.315	24.790	33.839	22.311	37.223
	*t*_1_	1	31.14	27.800	34.477	25.020	37.925	33.746	29.222	38.271	26.299	42.098
		2	36.99	33.648	40.325	30.283	44.358	39.594	35.070	44.119	31.563	48.530

**Table 12:** Bayesian point predictor with 95% and 99% ET prediction intervals for *Y*_*s*:10_ for *s* = 1, ⋯, 10.

Sch.	*s*	95%					99%				
		${\hat{Y}}_{s:10}$	IP		NIP		${\hat{Y}}_{s:10}$	IP		NIP	
			LB	UB	LB	UB		LB	UB	LB	UB
1	1	1.225	0.629	2.026	0.389	3.037	1.343	0.484	2.185	0.231	3.694
	2	1.573	0.740	3.088	0.479	5.541	2.532	0.600	3.665	0.310	8.146
	3	2.438	0.873	5.082	0.591	11.350	7.103	0.744	6.832	0.417	21.238
	4	4.613	1.018	8.538	0.720	23.780	19.710	0.906	13.182	0.548	57.920
	5	12.188	1.193	16.670	0.881	62.358	59.551	1.105	30.852	0.720	214.386
	6	32.653	1.382	34.263	1.062	174.841	151.749	1.320	77.551	0.921	878.949
	7	111.072	1.633	96.664	1.290	789.276	431.175	1.595	290.979	1.181	6816.226
	8	322.752	1.956	311.634	1.536	4.3E+03	1.0E+03	1.940	1.3E+03	1.467	6.9E+04
	9	1.4E+03	2.547	2.9E+03	1.856	4.4E+03	3.3E+03	2.570	2.2E+04	1.839	6.0E+06
	10	4.8E+03	3.582	5.6E+04	2.504	5.7E+04	8.6E+03	3.683	9.3E+05	2.497	6.2E+06

2	1	1.206	0.700	1.860	0.484	2.545	1.187	0.598	1.908	0.363	2.732
	2	1.431	0.797	2.612	0.566	4.036	1.454	0.698	2.782	0.441	4.653
	3	1.793	0.913	3.885	0.667	6.960	1.995	0.819	4.345	0.539	8.782
	4	2.373	1.040	5.853	0.780	12.137	3.163	0.954	6.914	0.653	16.897
	5	3.790	1.194	9.924	0.921	25.074	6.966	1.120	12.597	0.799	39.717
	6	7.234	1.362	17.479	1.079	54.221	17.287	1.302	24.036	0.966	99.035
	7	21.806	1.586	39.621	1.279	168.944	59.018	1.538	61.060	1.184	378.186
	8	69.039	1.873	99.508	1.502	599.893	179.077	1.833	174.902	1.430	1.7E+03
	9	427.945	2.388	591.669	1.803	7.7E+03	881.013	2.358	1.3E+03	1.766	3.3E+04
	10	2.0E+03	3.269	6.2E+03	2.135	8.0E+03	3.3E+03	3.257	1.9E+04	2.139	3.5E+04

3	1	1.200	0.764	1.733	0.565	2.238	1.180	0.686	1.743	0.467	2.303
	2	1.379	0.851	2.295	0.642	3.258	1.367	0.775	2.348	0.542	3.471
	3	1.641	0.953	3.184	0.734	5.067	1.656	0.880	3.334	0.633	5.649
	4	2.000	1.063	4.458	0.835	7.939	2.094	0.995	4.793	0.735	9.305
	5	2.660	1.195	6.877	0.959	14.269	3.082	1.133	7.660	0.863	17.860
	6	3.871	1.338	10.937	1.096	26.567	5.320	0.261	12.676	0.261	35.781
	7	7.978	1.526	21.416	1.268	66.594	14.177	0.388	26.261	0.328	99.524
	8	20.791	1.762	45.575	1.457	185.146	41.922	0.262	59.676	0.262	312.094
	9	135.939	2.175	198.062	1.710	1.5E+03	250.632	2.118	291.317	8.937	3.1E+03
	10	7.5E+02	2.857	1.4E+03	1.992	1.5E+03	1.2E+03	2.783	2.4E+03	1.970	3.2E+03

4	1	1.200	0.758	1.744	0.562	2.250	1.179	0.681	1.753	0.467	2.306
	2	1.383	0.845	2.314	0.637	3.266	1.369	0.769	2.361	0.540	3.449
	3	1.650	0.947	3.213	0.728	5.058	1.654	0.874	3.347	0.629	5.550
	4	2.010	1.059	4.500	0.830	7.878	2.063	0.989	4.797	0.730	9.016
	5	2.651	1.195	6.943	0.954	14.051	2.896	1.131	7.634	0.857	16.999
	6	3.762	1.343	11.034	1.093	25.919	4.621	1.288	12.564	1.000	33.356
	7	3.762	1.343	11.034	1.093	25.919	11.211	1.491	25.852	1.186	90.282
	8	18.076	1.791	45.946	1.468	176.052	32.499	1.742	58.240	1.398	273.941
	9	121.989	2.232	200.630	1.740	1.4E+03	212.132	2.180	281.921	1.694	2.6E+03
	10	7.2E+02	2.969	1.4E+03	2.051	1.4E+03	1.1E+03	2.906	2.2E+03	2.035	2.7E+03

## Data Availability

The data used to support the findings of this study are included within the article.
